# Skill Movement Trajectory Recognition of Freestyle Skiing U-Shaped Field Based on Deep Learning and Multitarget Tracking Algorithm

**DOI:** 10.1155/2022/7992045

**Published:** 2022-08-12

**Authors:** Yang Song, Lefa Zhao

**Affiliations:** ^1^China Academy of Olympic Higher Studies, Beijing Sport University, Beijing 100084, Beijing, China; ^2^Sports Training Academy, Shenyang Sport University, Shenyang 110102, Liaoning, China; ^3^Department of General Education, Shenyang Sport University, Shenyang 110102, Liaoning, China

## Abstract

Freestyle skiing U-shaped field is a snow sport that uses double boards to perform a series of action skills in a U-shaped pool, which requires very high skills for athletes. In this era of deep learning, in order to develop a more scientific training method, this paper combines multitarget tracking algorithm and deep learning to conduct research in freestyle skiing U-shaped venue skills motion capture. Therefore, this paper combines the convolutional neural network and multitarget tracking algorithm in deep learning to study the human action recognition technology, and then uses the LSTM module to study the freestyle skiing U-shaped venue skills. Finally, this paper designs the training method of the action recognition algorithm of the freestyle U-shaped skiing skills multitarget tracking algorithm based on deep learning. This paper also designs multitarget tracking dataset experiments and model updating experiments. Based on the data of experimental analysis, the training method designed in this paper is optimized, and finally compared with the traditional training method. Compared with the traditional freestyle U-shaped skiing skills training method, the experimental results show that the training method of the freestyle U-shaped skiing skills multitarget tracking algorithm action recognition algorithm is based on deep learning designed in this paper and this improves the skill score by 14.48%. Most professional students are very satisfied with the training method designed in this paper.

## 1. Introduction

Action recognition is a popular research topic in computer vision, which refers to the automatic identification and classification of human actions in videos by computers. It is affected by a series of conditions such as body shape, camera angle, moving objects, and background. Action recognition is essentially a video classification task, where many techniques and methods are used from the fields of image recognition and text retrieval. Research on action cognition is valuable for development in video surveillance, human–computer interaction, and other fields.

With the continuous improvement of the modern competitive level and the increasingly intensified competition, the development level of special physical characteristics, which is one of the main components of competitive ability, is becoming more and more prominent in modern competitive sports. China's freestyle U-shaped skiing skills have achieved good results in international competitions, and the competitiveness of the players is also rapidly improving. It is expected that the Winter Olympics will become a favorable event for China to win gold medals. Research basic theories and methods to develop the physical strength of freestyle skiing U-shaped field skill athletes, seek the best physical training theory and practice mode, and make the athletes' physical training process more scientific, systematic, and optimized.

In recent years, techniques including machine learning and deep learning have gradually emerged, and deep neural networks are already a highly topical subject of investigation and have made progress in various fields such as computer vision. Being an overarching subset of deep neural networks, convolutional neural networks are commonly employed in areas such as videographic processing and phonological identification. Its emergence also offers a fresh response to the issue of identifying human movements that we study. Therefore, this paper combines the application of deep learning and multitarget tracking algorithm in freestyle U-skiing skills, which can allow athletes to train scientifically and effectively.

The innovation of this paper lies in the use of convolutional neural networks in deep learning, and then through the research on human action recognition technology. This paper combines the LSTM module and the freestyle skiing U-shaped field skills, and finally constructs the application of the multitarget tracking action recognition algorithm based on deep learning in the freestyle skiing U-shaped field skills. This paper also designs multitarget tracking dataset experiments and model update experiments to optimize the algorithm designed in this paper.

## 2. Related Work

Recent developments in machine learning, particularly deep learning, have facilitated the recognition, classification, and quantification of medical image models. Deep learning has been rapidly gaining ground as a frontier, boosting the capability of all kinds of pharmaceutical operations. Shen D described the fundamentals of deep learning approach and reflected on previous achievements in registration of images, detection of anatomical and cellular structures, division of organizations, computer-aided disease prevention, and remediation [1]. Although his research is very deep in the field of deep learning, the combination of multitarget tracking algorithms is not complete. Segmentation is among the hugely talked about themes in hyperspectral remote-sensing technology. Over the last 20 years, he has proposed many methods to tackle the challenge of categorizing hyperspectral data. However, most of these do not have deep features. Chen et al. originally presented the notion of deep learning into hyperspectral data classification [2]. With the construction of communicative processes as automatically encoded, Oshea and Hoydis has developed a fundamentally novel way of looking at the design of a communicative process as an accountable end-to-end re-building project, with the aim of collaboratively optimizing the transponder and receptor subcomponents in an unique transaction. He presented the implementation of convolutional neural networks on primitive IQ models for the purpose of moderating selection. It achieved reliable precision in contrast to conventional scenarios that depend on specialist characteristics [3]. The utility of statistical analytics in health informatics for the past decades has increased dramatically with the influx of multimodal data. This has also led to a heightened fascination with producing a more collaborative production of analytical, data-driven versions of machine learning-based models in health informatics. Deep learning is a technique based on artificial neural networks that have appeared over the last few years as a formidable machine learning instrument that offers the potential to revamp the inevitable future of artificial intelligence. Ravi et al. provides a systematic and state-of-the-art revision of applied studies on deep learning in health informatics, providing a strategic assessment of the relevant advantages and drawbacks of the technology and its implications for the future [4]. Delande et al. introduced the hypothesis and isolated stochastic population (HISP) filter, a combined multitarget inspection/tracking approach originated from a fairly modern scheme of generating random species approximation. HISP filters are designed for multiobject estimation problems where the data association between orbits and collected observations has a moderate degree of ambiguity. HISP filters have linear complexity related to the number of targets and observations [5]. The structure of incremental motion (SfM) technique has shown excellent utility cross several recent investigations. Nevertheless, accuracy and soundness persist as major setbacks associated with these techniques. In this contribution, Cui et al. proposes a novel method for augmentative SfM that surmounts these problems in a unified frame consisting of two iterative circuits [6]. The results were tested in a wide selection of particular situations in sports video, completing a multitarget motion and multitarget monitoring solution suitable for a wide selection of situations in sports video. Duan applies deep neural networks to motion video multitarget kinematic shading reduction and accurate tracing to enhance detection behavior. Following the determination of the objective box options, the tracker estimates the multitarget motion limits of the target movement video using an optic streaming approach based on the multitarget movement of the object in the interframe movement video. The probe initially sweeps each moving picture frames frame by frame and looks at subregions of simultaneously detected and learned frames frame by frame until the present instant is very similar to the objective to be pursued [7]. To sum up, most of the above literature are about deep learning, multitarget tracking algorithms, and motion trajectory recognition. However, its main focus is on deep learning. How to build a freestyle skiing U-shaped venue motion trajectory capture and recognition based on multitarget tracking algorithm and deep learning is the main key of this paper.

## 3. Application Method of Multitarget Tracking Algorithm Based on Deep Learning in Action Recognition

### 3.1. Deep Learning

Deep learning [8] is a trendy study track in the domain of machine learning over the latest years. Deep learning techniques have gained tremendous recognition success in areas such as robot science, mathematics, engineering, and other fields, promoting the research and development of artificial intelligence. Referring to the remarkable progress made by deep learning in the field of computer vision, the first thing to mention is the great success of deep learning in image recognition, especially in image classification tasks [9].  Figure 1 shows the application areas of deep learning.

With the invention of machine learning models such as Support Vector Machines [10] and Deep Neural Networks [11], many artificial intelligence tasks are mainly done in feature engineering. Feature engineering refers to the process of using domain-related knowledge to study the data feature representation that can maximize the performance of machine learning algorithms. That is, the process of transforming the original data into feature data, so that these feature data can express the original data well. Feature engineering plays a very important role in machine learning. In practical applications, it can be said that feature engineering is the key to the success of machine learning. In many important competitions in the fields of machine learning and data mining, the winning teams often do not use very cutting-edge algorithms or improve algorithms, but use classical methods recognized by academia and industry. They win because they use domain knowledge to perform better feature engineering.

A typical feature of deep learning compared to shallow learning is that training requires large training datasets. The collection of datasets is a large workload, usually using data expansion methods [12, 13]. For example, image data trimming operations, digital image enhancement operations to improve image quality, these operations can derive a variety of complex samples.

Because features have a great impact on classification results, extracting important features representing objects is an important part of recognition. Traditional feature extraction is manually extracted, and features are mainly selected based on experience and professional knowledge. Deep learning is to automatically extract features through autonomous learning, effectively strengthening the firmness of human action cognition. Now, there are many deep learning models such as Scalable Networks (DBN) and Collapsible Neural Networks (CNN).

Deep learning extracts features through multiple layers, and the effect of multilayer feature extraction is better than that of single-layer or shallow feature extraction. Each level extracts different features according to the scale of the level. The low level is handed over to the high level after extracting the feature map. The high-level extracts the feature map from the feature map provided by the low-level again and passes it to the other party to extract the most effective recognition and features that improve the recognition accuracy.  Figure 2 shows the application of deep learning.

Convolutional neural networks have been mainly applied to tasks such as identity separation, monitoring, and discrimination. Schematically, in a convolutional neural network, a convolutional level and a subsampling level could constitute a characteristic selector [14]. In the convolutional level, a mechanic referred to as a “partially accepted area” is employed. This mechanism signifies that the nociceptors are not attached to all the nociceptors in the adjoining stratum, but are instead attached locally. Second, one of the other characteristics of the net is that it shares weights. By shared weights, we mean using kernels of the same magnitude of volume. Additionally, resampling is a key characteristic. Resampling is also known as pollarding, and there are two frequently employed ways of doing this: average pollarding and maximum pollarding. Average pollarding refers to counting the elements shared by the template and maximum pollarding refers to taking the average of the elements covered by the pollarding template. Various permutations of these characteristics or regimes have served as the cornerstones of some of today's frequently employed structures of convolutional neural networks. The current mature convolutional neural networks mainly include CaffeNet, AlexNet, GoogleNet, VGG, and ResNet. Its structure is shown in Figure 3.

Convolution is a classic concept in image processing. Calculate the local area of the image by using a two-dimensional matrix and obtain the corresponding convolution value. The convolution kernel, called an image filter, is a square matrix with weights. Filters can be applied to image areas. It usually uses multiple filters simultaneously [10]. For example, apply a 6 × 6 filter to an image. Then, the pixel value of the output coordinate is the weighted sum of the 6 × 6 area of the input image, and the same can be said for other pixels. This operation makes the convolutional neural network very effective for the recognition of two-dimensional images.

In a convolutional layer, the input data are convolved with several filters. The result of applying a filter to an image is called a feature map, and the number of feature maps is the same as the number of filters. If the preapplicator layer is a convolutional layer, the filter is applied to the feature map. This is the same as inputting feature maps and outputting other feature maps. Intuitively, when the weights are spread over the whole image, the features do not depend on the location, and multiple filters can detect different features separately.

### 3.2. Human Action Recognition

The basic flow of the human action recognition algorithm is shown in Figure 4, and the specific steps are as follows:

1. Image preprocessing [15]. When inputting a single or a series of image data, first perform image-preprocessing operations such as framing, image resizing, image selection, image enhancement, and then pass the obtained image to the next step.
2. Detection of moving objects [16]. Moving object detection refers to segmenting human foreground objects from still images, or segmenting corresponding action sequences in image sequences, to obtain moving objects with a small amount of data and efficient information. There are two methods for segmentation of the human body domain. One is a method of segmenting the human body domain based on image segmentation. Another method is to combine the image segmentation method according to the human image model, and obtain the human body area by the method of image matching.
3. Feature extraction. After the human domain detection is completed, the next step is feature extraction. The purpose of feature extraction is to extract a part of feature information from a single or a series of image data, which is characterized by human behavior, and the features are extracted from previous experience. General static feature extraction methods include: Histogram of Oriented Gradients (HOG), Local Binary Patterns (LBP), and Haar-like feature methods. Common dynamic extraction methods include spatiotemporal interest point algorithm (STIP), histogram of directional optical flow (HOF), and moving boundary feature (MBH).
4. Analysis and identification of functions. After the feature extraction is completed, the obtained feature is a high-dimensional feature vector. In order to realize the classification of human actions, the feature vector needs to be analyzed. Commonly used feature analysis methods include human body model-based feature understanding and statistical model-based feature understanding. Among them, the human body model-based feature understanding method obtains results by comparing the obtained human action performance with existing action models. The feature understanding method based on statistical model establishes the feature data template of each action, compares the acquired feature data with the action template, and calculates the similarity to determine the action type. According to the above steps, the classification results of human actions can be completely obtained.

### 3.3. SSD Target Detection

The SSD model [17] is an end-to-end object detection method like the YOLO model. Unlike YOLO, SSD discretizes the space of the predicted bounding box output into a set of default boxes. During detection, a score is predicted for the category of each object that appears in each default box, and the size of the detected bounding box is rescaled to better match the detected object.

SSD methods mainly use a series of small convolutional filters to predict class scores and position offsets for a fixed set of default bounding boxes on feature maps. . Generate predictions at various scales from feature maps at different scales and correctly predict various aspect ratios. The detection speed of SSD is almost as fast as YOLO, and it is as accurate as the detection method using region proposal technology and ROI pooling. The principle of SSD target detection is shown in Figure 5.

The SSD model approach is also based on a feedforward neural network that integrates all computation, feature extraction, detection, and normalization processes into one network. The network structure of the SSD model is shown in Figure 6. The VG16-SSD network, a standard network for image classification, is used. The basic features are extracted using the basic network of the model, and several auxiliary structural layers and convolutional layers are added after the basic network to generate the final detection target on the left and the multiscale features corrected by the bounding box. Auxiliary convolutional layers, in different network layers, extract a fixed-size set of bounding boxes and predict a score for the class of objects in all bounding boxes. Finally, the nonmaximum suppression algorithm is used to propose the redundant frame to generate the final detection result.

As shown in the figure, when the SSD network is trained for detection, six feature layers are extracted as the final detection features, and the scale of these feature maps is gradually reduced, so that multiscale features can be extracted and the final detection results are more accurate. Applying a set of convolutional filters to each feature layer produces a corresponding fixed-size prediction.

### 3.4. Forward and Backward Processing of LSTM Module

Like ordinary recurrent neural networks, LSTM networks are trained using the BPTT method [18], and the partial derivatives of model parameters are calculated and updated through two forward and backward processing processes. Before discussing the forward and backward processing of LSTM network in detail, we first define several concepts unique to the LSTM module. Let the subscripts *γ*, *θ*, and *ω* denote the input gate, the forgetting gate and the output gate, respectively, and the subscript *h* denotes the input of the LSTM module. Without loss of generality, it is assumed here that an LSTM module contains only one internal state *Z*. The LSTM network also processes a sequence *a* of length *S*, the forward operation starts at *s* = 1, and the backward operation starts at *s* = *S*.

Forgotten gate:

(1) $$\begin{array}{c} u_{\theta }^{s}=\sum_{i=1}^{I}w_{i\theta }a_{i}^{s}+\sum_{h=1}^{H}w_{h\theta }a_{h}^{s-1}+w_{z\theta }Z^{s-1},\\ a_{\theta }^{s}=f_{\theta }\left(u_{\theta }^{s}\right). \end{array}$$

Input gate:

(2) $$\begin{array}{c} u_{\gamma }^{s}=\sum_{i=1}^{I}w_{i\gamma }a_{i}^{s}+\sum_{h=1}^{H}w_{h\gamma }a_{h}^{s-1}+w_{z\gamma }Z^{s-1},\\ a_{\gamma }^{s}=f_{\gamma }\left(u_{\gamma }^{s}\right). \end{array}$$

Internal state:

(3) $$\begin{array}{c} u_{z}^{s}=\sum_{i=1}^{I}w_{iz}a_{i}^{s}+\sum_{h=1}^{H}w_{hz}a_{h}^{s-1},\\ Z^{s}=a_{\theta }^{s}Z^{s-1}+a_{\gamma }^{s}f_{z}\left(u_{z}^{s}\right). \end{array}$$

Output gate:

(4) $$\begin{array}{c} u_{\omega }^{s}=\sum_{i=1}^{I}w_{i\omega }a_{i}^{s}+\sum_{h=1}^{H}w_{h\omega }a_{h}^{s-1}+w_{z\omega }Z^{s},\\ a_{\omega }^{s}=f_{\omega }\left(u_{\omega }^{s}\right). \end{array}$$

Status output:

(5) $$\begin{array}{c} a_{h}^{s}=a_{\omega }^{s}f_{o}\left(Z^{s}\right). \end{array}$$

Similarly, it is not difficult to derive the backward processing process of LSTM recurrent neural network according to the BPTT method. Here, the definitions of the two quantities are given as follows: the backward processing process of the LSTM network on the state output, output gate, internal state, forget gate, and input gate, respectively, is given.

(6) $$\begin{array}{c} \epsilon_{o}^{s}≜\frac{\partial J}{\partial a_{h}^{s}},\\ \epsilon_{o}^{s}≜\frac{\partial J}{\partial Z^{s}}. \end{array}$$

Status output:

(7) $$\begin{array}{c} \epsilon_{o}^{s}=\sum_{k=1}^{K}w_{zk}\delta_{k}^{s}+\sum_{h=1}^{H}w_{zh}\delta_{h}^{s-1}. \end{array}$$

Output gate:

(8) $$\begin{array}{c} \delta_{\omega }^{s}=f_{\omega }^{\prime }\left(u_{\omega }^{s}\right)f_{o}\left(Z^{s}\right)\epsilon_{o}^{s}. \end{array}$$

Internal state:

(9) $$\begin{array}{c} \epsilon_{z}^{s}=a_{\omega }^{s}f_{o}^{\prime }\left(Z^{s}\right)\epsilon_{o}^{s}+a_{\theta }^{s+1}\epsilon_{z}^{s+1}+w_{z\gamma }\delta_{\gamma }^{s+1}+w_{z\theta }\delta_{\theta }^{s+1}+w_{z\omega }\delta_{\omega }^{s},\\ \delta_{z}^{s}=a_{\gamma }^{s}f_{z}^{\prime }\left(u_{z}^{s}\right)\epsilon_{z}^{s}. \end{array}$$

Forgotten gate:

(10) $$\begin{array}{c} \delta_{\theta }^{s}=f_{\theta }^{\prime }\left(u_{\theta }^{s}\right)Z^{s-1}\epsilon_{z}^{s}. \end{array}$$

Input gate:

(11) $$\begin{array}{c} \delta_{\gamma }^{s}=f_{\gamma }^{\prime }\left(u_{\gamma }^{s}\right)f_{\text{z}}\left(u_{\text{z}}^{s}\right)\epsilon_{z}^{s}. \end{array}$$

Sports model:

(12) $$\begin{array}{c} Azz_{s}^{k}=\frac{\left(Z_{s}^{k}-Z_{s-1}^{j}\right)-\left(Z_{s-1}^{j}-Z_{s-2}^{i}\right)}{\Delta S^{2}},\\ V_{s}^{k}=\frac{Z_{s}^{k}-Z_{s-1}^{j}}{\Delta S}+Azz_{s}^{k}\times \Delta S,\\ {\hat{Z}}_{s+1}^{*}=Z_{s}^{k}+V_{s}^{k}\times \Delta S+\frac{Azz_{s}^{k}\times {\left(\Delta S\right)}^{2}}{2}. \end{array}$$

### 3.5. Freestyle Skiing U-Shaped Venue Skills

In the U-shaped field competition of freestyle skiing [19], on the U-shaped field with a length of 100 to 150 m, a width of 13 to 17 m, a depth of 4 to 6 m, and an inclination of 15 to 20°, various aerial skills can be displayed. Athletes' various technical movements, sliding, and rotations in the “U”-shaped groove require a high degree of balance, flexibility, and inherent receptive ability of the athlete's neural process to decelerate and take off with the help of the U-shaped groove. It hits the wall and completes difficult technical actions such as flying in the air, grabbing, and turning. The freestyle skiing U-shaped skill event is a favorable event for China. In the recent 2022 Winter Olympics, Gu Ailing's gold medal in the event laid a solid foundation for the next Milan-Cortina 2026 Winter Olympics. China will continue to work hard to prepare for the next event. Therefore, the scientific research of this project has continued to deepen in recent years. In free-skiing u-court competitions, if the athlete has the same score in the single jump competition, it is determined by the highest height score in the action set. Athletes' core muscles can achieve a higher height. In addition to that, the height will be reduced. In addition, because a complete set of jumps and twists is also key to high competitive scores, most athletes in various countries train with these two sports as the focus of their training.

The stage of the U-shaped field is divided into two stages. One is the U-shaped ski field and the stage where the action is done in the air. The stage where the action is done in the air mostly reflects the athlete's somersault. The sliding stage of the swivel-capable field on the U-shaped ski resort covers the athlete's take-off and landing control ability. For take-off, speed and take-off angle are the two most direct physical parameters, because the athlete obtains the ideal height to complete high-quality movement, so choosing the most reasonable take-off angle as the premise of a specific speed is the core issue. The secret to a successful landing is to control the body with a certain initial speed as the premise, and at the same time to achieve high-quality movement, enter the U-shaped field again and land successfully. This stage is the way to maintain speed and balance. On the U-shaped ski field, athletes can reasonably use the sliding speed of the accelerated slope to perform somersaults, twists, swings and various action switching functions. The most obvious performance feature of this technique is the difficulty of the athlete's movement, the completion of the movement flight height, and the aerial movement posture.

#### 3.5.1. Speed Characteristics

The freestyle U-shaped track skier obtains the height of entering the groove through the acceleration sliding of the landslide, from the initial acceleration of the landslide until entering the U-shaped groove, that is, the kinetic energy is converted into the gravitational potential energy. During the take-off process in the slot, the kinetic energy is converted into gravitational potential energy, while the gravitational potential energy decreases and the kinetic energy increases during the falling process. The sliding speed determines the slotting angle of different action techniques. The perfect application of the speed lies in the precise control of the athlete in the sliding, and its speed characteristic is embodied as “steady.”

#### 3.5.2. Slotting Angle Features

In the 5–6 take-off movements of freestyle U-shaped skiers in the groove, different movement techniques have different out-of-the-groove angles. The slotting angle determines the landing area of the action, and the correctness of the landing zone directly affects the success or failure of a single action, so the slotting angle is characterized as “accurate.”

#### 3.5.3. Flight Altitude Characteristics

If freestyle U-shaped skiers do not have good sliding ability, they will not have high-quality take-off speed, which will affect the flying height and the completion of high-quality difficult movements. Therefore, the flight altitude characteristic of this project is expressed as “high.”

#### 3.5.4. Action Technical Characteristics

In the complete set of movements of the freestyle U-shaped field skiing project, there must be a basic movement in the rules, and then the smoothness of the connection between the movements, and the application of the difficulty of the movements. When other factors are satisfied, the use of action difficulty determines the final success or failure of the game, and its action difficulty characteristics are embodied as “beautiful” and “difficult.”

## 4. Tracking Algorithm Dataset Evaluation Experiment

### 4.1. Single-Target Tracking Dataset Experiment

This paper uses OTB100 for the assessment of the dataset. OTB100 consists of a grand total of one hundred recorded tracking video clips, which are integrated from various datasets. The evaluation mark uses one-pass valuation (OPE) profile as an assessment indicator. By definition, the OPE profile is the outcome of just a single trace, that is, the current tracking chain is ended when the tracking fails, and no reinitialization is necessary. The OPE profile has two types of assessment, as shown in Figure 7, one of which is based on the area overlap rate. A frame is deemed to be correctly followed when the area of the algorithm's prediction and the estimated area of the commented frame overlap by more than a specified amount. The total number of consecutive completed frames as a percentage of all frames is called the success rate. The other type of evaluation is predicated on patient offsets [20, 21]. A frame is deemed to be correctly followed when the deviation between the perimeter of the frame forecast by the operator and the epicentre of the tagged frame of a particular frame is smaller than a certain threshold. The proportion of overall completed frames to all frames is referred to as accuracy. These two curves supplement each other and one cannot be used without the other. For instance, a percent of success can assess the variability in target dimensions, but not accuracy. The score of the surface area of the profile is the primary indicator of assessment.

The selection of traditional correlation filter-based individual objective pursuit algorithms is presented in this chapter and compared with deep learning-based individual objective pursuit algorithms, as shown in Table 1 [22]. Among them, MDnet is far ahead of other algorithms in terms of success rate and accuracy rate. GOTURN is the fastest, but has the worst effect among many algorithms. The SiameseFC network balances MDNet and GOTURN, and the effect is greatly improved compared to GOTURN, but the speed is doubled. Although the speed of Siamese is not as good as that of GOTURN, it still far exceeds the speed of other algorithms. Compared with other traditional single-target tracking algorithms, discriminative scale space tracking (DSST), multiple entropy minimization (MEEM), the channel and space based discriminative correlation filter (CSR-DCF), and the effects of deep learning-based individual objective pursuit algorithms are highly competitive in some respects (success rate, accuracy and speed) [23, 24].

### 4.2. Multitarget Tracking Dataset Experiment

MOT2015 is a multiobject tracking dataset containing 22 video sequences. The collection devices include both stationary and mobile camcorders, and the acquisition views consist of elevated, overhead, and downward views, as well as varying meteorological situations and varying illumination requirements. The video sequence has 11286 images, of which the control collection consists of 5500 images, 500 objects, and 39,905 frames. The training session consisted of 5500 images with 721 tracking targets and 61440 tracking target frames. The dataset offers inspection frames gained from fused passage characteristics (ACF). The specific distribution of the data is shown in Tables 2 and 3.

Among them, the detector of MOT2016 is replaced by a deformable component model (DPM), which has a higher target localization accuracy than the fusion channel feature detector used in MOT2015. So in general, the same algorithm, the indicators on MOT2016 will be slightly higher than the results on MOT2015. The annotation files of MOT2015 and MOT2016 are also different. MOT2015 provides the 3D information of the target, but only labels people. MOT2016 not only abandons 3D information but also labels cars, bicycles, motorcycles, etc. The specific distribution of the data is shown in Tables 4 and 5. The results are shown in Figure 8.

A simple comparison shows that STAM has fewer missed detections (FN) and label switching (IDSw), but more false detections (FP) when the overall effect (MOTA) is not much different. STAM and AMIR, respectively, represent the idea of two different multitarget tracking algorithms. Among them, STAM can retrieve the lost target by constructing a matching convolutional neural network, that is, less missed detection. However, due to the algorithm itself, the missed detections retrieved may not be correct, so more false detections are brought about. AMIR can eliminate a large number of false detections by building an association model based on recurrent neural network, but there is no way to make up for lost targets [25, 26].

### 4.3. Model Online Update Test Experiment

The two most important parts of the tracking process are the tracking strategy for the model. After initializing the parameters of the network model by a certain method, the input of the first frame can be accepted to predict and locate the target object in the subsequent frames. However, during the tracking process, the target object is constantly changing, and will experience deformation, occlusion, blurring, etc., resulting in a larger and larger difference between the target object and the initial state. The ability of the initial model to fit the features of the target object decreases. If the model is not updated according to the latest state sampling of the target object, the target will be transferred or lost. The subject has been tested, and the experimental results of the test model fixed and online update in the OTB2015 data set are shown in Figure 9.

It can be seen from the experimental results of the graph that the accuracy and success rate of the algorithm are higher than those when the model parameters are fixed when the model is updated.

## 5. Application Analysis of Multitarget Tracking Algorithm Based on Deep Learning in Freestyle U-Shaped Ski Resorts for Action Recognition

Through the test of the data set, the action recognition algorithm of the freestyle U-shaped skiing skill multitarget tracking algorithm based on deep learning designed in this paper is optimized [27]. In order to verify the effect of the optimized algorithm on the freestyle U-shaped ski field, a set of control experiments was designed in this paper, with 10 people in each group. One group was trained using the deep learning-based freestyle U-ski skill multitarget tracking algorithm action recognition algorithm designed in this paper, and the other group was trained using traditional training methods. Finally, by judging the improvement of its skill scores and the personal feelings of 50 professional students, the advantages of the multitarget tracking algorithm for freestyle U-shaped skiing skills designed in this paper based on deep learning are judged. The experimental results are shown in Figure 10.

As can be seen from the figure, the skill score of the multitarget tracking algorithm for freestyle U-shaped skiing skills based on deep learning designed in this paper after the training of the action recognition algorithm reached 92.96 points. The freestyle U-shaped skiing skills based on traditional training methods scored only 81.2 points. This shows that the training method of the multitarget tracking algorithm for freestyle U-shaped skiing skills based on deep learning designed in this paper improves the skill score by 14.48% compared with the traditional method. Moreover, 27 people were very satisfied with the training method of the multitarget tracking algorithm action recognition algorithm for freestyle U-shaped skiing skills based on deep learning designed in this paper, and 13 people were quite satisfied with this training method. This shows that the training method of the multitarget tracking algorithm for freestyle U-shaped skiing skills based on deep learning designed in this paper has a great improvement compared with the traditional training method and is very popular among professional students.

## 6. Conclusion

This paper mainly studies the application of skill motion capture technology combined with multitarget tracking algorithm in the U-shaped field of freestyle skiing under the background of deep learning. Therefore, this paper combines the research of convolutional neural network in deep learning with multitarget tracking algorithm, and then selects the LSTM module to study the U-shaped field skills of freestyle skiing in the context of human action recognition technology. Finally, this paper designs a training method for the action recognition algorithm of freestyle U-shaped skiing skills multitarget tracking algorithm based on deep learning. Then this paper designs a multitarget tracking data set experiment, analyzes the data set, and improves the algorithm based on the results of the data set analysis. Then this paper updates the model locally through model update experiments. Finally, this paper uses experiments to verify the role of the training method of the deep learning-based freestyle U-shaped skiing skills multitarget tracking algorithm action recognition algorithm in professional students.

## Figures and Tables

**Figure 1:** Application areas of deep learning.

**Figure 2:** Application of deep learning.

**Figure 3:** The structure of the convolutional neural network.

**Figure 4:** Flowchart of traditional action recognition.

**Figure 5:** Flow chart of SSD model detection.

**Figure 6:** SSD network structure diagram.

**Figure 7:** The results of the single target tracking algorithm on the OTB100 dataset.

**Figure 8:** STAM and AMIR test results in MOT2016: (a) STAM results on the MOT2016 test subset. (b) AMIR results on the MOT2016 test subset.

**Figure 9:** Comparison of model fixed and new update experiments.

**Figure 10:** Comparison of experimental results: (a) Skill score comparison. (b) Satisfaction evaluation.

**Table 1:** Comparison of single target tracking algorithms.

Algorithm	MDNet	SiameseFC	GOTURN	DSST	MEEM	CSR-DCF
Success rate	0.675	0.582	0.445	0.52	0.53	0.598
Accuracy	0.903	0.771	0.572	0.693	0.781	0.733
Speed (fps)	1	70	165	24	10	13

**Table 2:** MOT2015 training set data statistics.

Name	Frame rate	Resolution	Length (frame)	Target (s)	Detection frame (units)	Density (units)
ADL-Rundle-6	30	1920 × 1080	525	24	5009	9.5
ADL-Rundle-8	30	1920 × 1080	654	28	6783	10.4
KITTI-I3	10	1242 × 375	340	42	762	2.2
KITTI-17	10	1242 × 370	145	9	683	4.7
Venice-2	30	1920 × 1080	600	26	7141	11.9

**Table 3:** MOT2015 test set data statistics.

Name	Frame rate	Resolution	Length (frame)	Target (s)	Detection frame (units)	Density (units)
ADL-Rundle-1	30	1920 × 1080	500	32	9306	18.6
ADL-Rundle-3	30	1920 × 1080	625	44	10166	16.3
KITTI-16	10	1242 × 370	209	I7	1701	8.1
KITTI-19	10	1242 × 374	1059	62	5343	5.0
Venice-1	30	1920 × 1080	450	17	4563	10.1

**Table 4:** MOT2016 training set data statistics.

Name	Frame rate	Resolution	Length (frame)	Target (s)	Detection frame (units)	Density (units)
MOT16-02	30	1920 × 1080	600	49	17833	29.7
MOT16-04	30	1920 × 1080	1050	80	47557	45.3
MOT16-05	14	640 × 480	837	124	6818	8.1
MOT16-09	30	1920 × 1080	525	25	5257	10.0
MOT16-10	30	1920 × 1080	654	54	12318	18.8

**Table 5:** MOT2016 test set data statistics.

Name	Frame rate	Resolution	Length (frame)	Target (s)	Detection frame (units)	Density (units)
MOT16-01	30	1920 × 1080	450	23	6395	14.2
MOT16-03	30	1920 × 1080	1500	148	104556	69.7
MOT16-06	14	640 × 480	1194	217	11538	9.7
MOT16-07	30	1920 × 1080	500	55	16322	32.6
MOT16-08	30	1920 × 1080	625	63	16737	26.8

## Data Availability

Data sharing is not applicable to this article as no new data were created or analyzed in this study.
